# The Role of an Exoskeleton Simulation of Senescence in Health Sciences Education

**DOI:** 10.1155/2023/3148896

**Published:** 2023-05-29

**Authors:** Rodrigo Ramos-Zúñiga, Jorge A. González-Rios

**Affiliations:** Translational Neurosciences Institute, University Center of Health Sciences, University of Guadalajara, Guadalajara, Jalisco, Mexico

## Abstract

**Background:**

Education in the formation of human capital in health constantly presents challenges. New tools in the emerging contexts may strengthen empathic attitudes. We developed an educational intervention that included a senescence simulator and assessed its impact on perception and attitudes in healthcare students.

**Methods:**

A cross-sectional comparative study was conducted that assessed acquired knowledge and self-perception using a semistructured survey administered before and after the demonstration and intervention using the simulator and reported the experience through the role of the patient and caregiver. The data were analyzed statistically to identify the demographic characteristics and differences between the groups of students. The data were analyzed statistically to identify the demographic characteristics and differences between the groups of students in the responses pre-post intervention, using statistical software (IBM SPSS Statistics 26.0).

**Results:**

Of the 256 participants surveyed before the intervention, 93.8% described cognitive deterioration as a significant disability and 53.1% considered the health system to be inadequate in meeting the needs of older individuals. Only 59.8% stated that the current academic training meets the educational requirements for the care of the elderly. In total, 98.9% of the participants reported that the simulator changed their perception by increasing their empathy. In total, 76.2% showed greater sensitivity to older adults and 79.3% reported that the experiential learning consolidated their professionalizing perspective. Among the younger participants (aged 18–20 years), sensitivity and reorientation toward pursuing an associated graduate degree were higher after the intervention (*p*=0.01).

**Conclusions:**

Educational strategies, such as the senescence simulator, offer an experiential intervention that strengthens the knowledge and attitudes toward older individuals. During the pandemic emergency, it proved to be a useful educational strategy in consolidating caring behavior as a hybrid educational tactic. The senescence simulation enabled the participants to widen their educational and professional schemes to encompass the care of the older population.

## 1. Introduction

Senescence, a physiological process that affects living beings, involves different homeostatic mechanisms at the cell level, tissue atrophy, and subsequent decreased function, thereby increasing the risk of comorbidities and their complications [1–5].

According to the estimations by the World Health Organization (WHO, 2021), older adults will reach a ratio of 1 : 6 people in 2030 [6], and by 2050, the number of adults older than 60 years will be twice as high (2.1 billion) [7, 8]. Therefore, the future demand for the care of older adults imposes significant challenges for the healthcare system given its increase, mainly due to demographic transition and the fact that older people are the primary health service and budget consumers [9–12].

This demographic transition leads to an epidemiological transition and represents an impact on public health that should strengthen health sciences education programs and curricula. Traditional methods are informative and situational in nature, but until recently, experiential strategies have gradually been incorporated that allow us to perceive, through different sensory modalities, everything that happens to the older adult patient. In different studies and educational contexts in health sciences, this contributes not only to consolidating learning but also to generating greater sensitivity in the approach of health service users.

Different examples applied to students of medicine, pharmacy, and especially nursing show the potential outcome of these tools on the quality of care for adults in the geriatric area.

As stated in previous studies, stimulating empathic behaviors through pedagogic innovations has a bigger impact on education than the use of traditional models and results in a significant learning process. Today, the use of the simulator represents a unique experience for medical, nursing, physical, and cognitive rehabilitation trainees and for all professionals who care for older adults, which can generate changes towards a more tolerant and compassionate behavior in the care of patients with chronic diseases or geriatric patients [13–15].

The use of simulation strategies can be linked to a higher quality of basic geriatric care and strengthen the educational orientation of future professionals towards this segment of an increasingly ageing population [16–20]. Such is the case of new technological resources for education such as simulator actors, high and low fidelity mannequin simulators, virtual reality, gamification, and metaverse, which are supported by the pedagogy of cognitive-behaviorism, constructivism, and connectivism [21, 22].

In the present study, we developed a learning strategy to assess its effect on the educational perception of health science students. This was achieved by employing an informative scientific educational program regarding senescence and the use of exoskeleton simulating senescence. Under specific situational circumstances, *in vivo* was used in order to identify and test the most common functional limitations of the geriatric patient (presbyopia, presbycusis, coordination deficits, extrapyramidal tremor, degenerative osteoarthrosis, stiffness, bradykinesia, stiffness, bradykinesia, alterations in postural balance, sensory changes resembling neuropathy and radiculopathy, and resting tremor through an electric stimulator that mimics the involuntary movement of Parkinson's disease and limits voluntary movements such as writing). We aimed to identify the role of this intervention in the generation of stronger bonds with the students' emotional and cognitive attitudes towards the elderly [23–25].

## 2. Materials and Methods

This cross-sectional comparative quasi-experimental educative intervention study assessed the impact of an educational intervention, which constituted a purposefully developed senescence simulator designed for us by a quasi-experiment trial. The intervention was presented in scheduled sessions to randomly selected representative groups of students pursuing different professional fields of health sciences from March to June 2021, in Guadalajara, Mexico, at the University of Guadalajara, the second most largest public university in the country.

Although the selection of representative groups was random, at least one group from each degree course and discipline was selected freely upon formal invitation by their course teachers. The dynamics consisted of the application of a preassessment via Google form *in situ*, followed by a brief slide presentation with information related to senescence and physiological changes due to age and a demonstrative video and then a volunteer carrying all the elements of the exoskeleton with the help of an assistant who would represent the role of the caregiver. The scenario involved performing some basic tasks such as walking, sitting, standing, climbing stairs, picking up fine objects, and signing a document. Afterwards, the postassessment was applied to all participants through the Google form platform, and the event was concluded. The estimated time of the whole process was 30 minutes.

The preintervention and postintervention surveys comprised 11 and 7 questions, respectively. The surveys included multiple choice and closed-ended questions based on a Likert's 5-score scale [26]. The collected data were statistically analyzed to identify demographic data and differences between the groups, as well as the differences before and after the intervention.

For the statistical analysis, SPSS version 26.0 (IBM TM) software was used for basic demographic data such as age, gender, and occupation and for the comparative analysis of groups to identify differences in the preintervention and postintervention surveys that were statistically significant at *p* < 0.05 in the contingency table. Chi-square (exploration of significance data) and Fisher's test (confirmation of significant value) were applied for the analysis of presurvey and postsurvey, knowledge of adult disabilities, and analysis of responses by gender, age, and degree, and the results are presented that represented an impact under statistically significant evidence.

This study was assessed and approved by the Research Ethics Committee under record DGRPID/DI/CEI/15/21. It was conducted pursuant to the rules of the institution and national regulations, such as the “Mexican General Health Law on Research,” and classified as a riskless study for participants. In all cases, informed consent was obtained, and the data provided were anonymous and confidential. Only video tutorial participants authorized the use of their image in the demonstration video. The tutorial type video was developed by us with professional technical support and was designed according to the contents with the participation of teachers and students with previous training for the demonstration of the use of the simulator. It was presented in native language (Spanish) and was identified with a pilot plan that represented coherence and validity with the objectives of the protocol and correlation with the survey questions (https://youtu.be/vprn3fXmBDA).

### 2.1. Design and Background

The strategy was applied *in situ* in the classroom of each group studied. In some groups, due to the pandemic, a prerecorded tutorial video was sent with all the dynamics of the application of the exoskeleton and the tasks to be carried out as introductory information, and the application in real time was only presented to 50% of each group in presential form. Those who participated in the tutorial video recording were students who collaborated on a voluntary basis under direct invitation. All participants were from a single health sciences institution of the University of Guadalajara who were recruited directly by invitation through their professors, after a random selection according to professional fields and school schedules. This strategy is not a formal part of its curricular design and was presented as an alternative practice with voluntary and open participation.

The methodological strategy constituted the application of the preintervention and postintervention surveys as part of the evaluation of senescence-related educational content as well as the experiential use of the exoskeleton (Figure 1). Half of the health science students carried the simulator to experience the different physical disabilities present in the elderly, while the other half participated in the role of caregiver to carry out the different activities proposed.

The educational tutorial preintervention was conducted with online instructions using Google with the groups of students pursuing different health science degrees, including medicine, nursing, nutrition, physical education and sports, psychology, and radiology. The inclusion criteria were pursuing a degree associated with health sciences and be an active regular student or higher degree at the time of the survey. The exclusion criteria of the study were oriented to students who did not participate in both the surveys and those who were not pursuing a degree in the field of biomedical sciences at the time of taking the surveys.

### 2.2. Study Variables

The main dependent variables were (1) change in perception and understanding toward the physical and cognitive limitations of older individuals, (2) generation of a positive impact on professionalism to provide better care for older individuals, and (3) reevaluation of the decision to pursue a specialized or graduate degree oriented toward the care of older people. The independent variables included the application of the educational intervention and reinforcement of knowledge that involved the use of an exoskeleton simulating physical senescence.

### 2.3. Statistical Analysis

Statistical Package for the Social Sciences (SPSS IBM) software was used for the statistical analysis of the study data (age, gender, and occupation). Central tendency measures were analyzed for demographic data, and chi-square, Fisher's exact, and Student's *t*-tests were used to identify the statistical significance between the groups, considering a ^*∗*^*p* < 0.05 with a *p* value estimated for contingency tables. Chi-square (exploration of significance data) and Fisher's test (confirmation of significant value) were applied for the analysis of presurvey and postsurvey, knowledge of adult disabilities, analysis of responses by gender, age, and degree, and results with a statistically significant impact are presented.

## 3. Results

In total, 294 and 282 responses were obtained from the preintervention and postintervention surveys, of which 38 and 26 responses were excluded due to the exclusion criteria, respectively.

### 3.1. Participants' Demographic Data

The mean age of the participants was 21 years (interquartile range = 2), and 78 of them (30.5%) were male. In terms of the study area, 13 students (5.1%) were from physical education and sport, 65 (25.4%) from nursing, 82 (32%) from medicine, 23 (9%) from nutrition, 61 (23.8%) from psychology, and 12 (4.7%) from radiology.

### 3.2. Care Scenario for Older Individuals before the Intervention

In the preintervention period, a total of 216 (84.4%) participants planned to pursue a specialized or graduate degree and 38 (14.8%) considered it a possibility. Moreover, when presented with a hypothetical situation, only 27 participants (10.5%) considered the possibility of pursuing a specialized or graduate degree oriented toward the care of older people, 77 (30.1%) chose pediatric care, 31 (12.1%) chose adolescence care, and 121 (47.3%) chose adult care.

Overall, 141 (55.1%) participants reported having cared for an older adult and 70 (27.3%) participants were familiar with the approximate fall rate in this population, whereas 79 (30.9%) were not. Regarding knowledge of the main disabilities among older adults, cognitive deterioration was noteworthy since 240 (93.8%) of the participants mentioned this disability, followed by osteoporosis and cataracts mentioned by 223 (87.1%) and 216 (84.4%) participants, respectively. The complete results are summarized in Table 1.

The perception of whether the current health system adequately meets the needs of this population yielded the following results based on Likert's scale: 67 (26.2%) participants answered neutrally and 136 (53.1%) disagreed.

Regarding training to manage and meet the needs of the older population and whether such training is adequate, 84 (32.8%) of the participants considered it adequate and totally agreed, whereas 46 (18%) simply agreed. Finally, 142 (55.5%) participants reported that the biggest social concern that older adults face is abandonment, followed by intolerance, discrimination, and violence as reported by 92 (35.9%), 12 (4.7%), and 10 (3.9%) participants, respectively (Table 1).

### 3.3. Perception of Older Adults' Surroundings after the Intervention

After the educational intervention, the participants were administered a second survey that evaluated the knowledge and self-perception awareness acquired by the students due to the intervention. Only 32 (12.5%) participants were familiar with all the limitations faced by the older population that were mentioned in the educational session, while 202 (78.9%) were only aware of a few and 22 (8.6%) were completely unaware of such limitations (Table 2).

The following questions were answered according to the 5-score Likert's scale model. When asked whether the intervention had altered their perception and empathy toward the older population, 195 participants (76.2%) totally agreed and 58 (22.7%) agreed. When asked whether the intervention positively affected their professionalism in providing better care to the older population, 203 participants (79.3%) totally agreed and 52 (20.3%) agreed. When the participants with prior experience in caring for older adults were asked if they would change the way they cared for the older population in the future, 142 (55.5%) totally agreed and 42 (16.4%) agreed.

Moreover, when the participants were asked whether they would reconsider pursuing a specialized or graduate degree associated with caring for older individuals, 37 participants (14.5%) totally agreed and 87 (34%) agreed.

When asked whether the education provided by the institution of the participants regarding older people care was adequate, 89 participants (34.8%) totally agreed and 64 (25%) agreed. Finally, 137 participants (53.5%) totally agreed and 94 (36.7%) agreed that the simulation-based exoskeleton was useful for health sciences education regarding the care of older individuals (Table 3).

Statistical analysis highlighted cognitive deterioration, osteoporosis, cataracts, and decreased motor skills as the most frequent signs observed in older individuals as identified by most of the participants of all age and degree groups.

In the preintervention survey, only 10.5% of the participants considered working in a professional activity associated with the older population (*p*=0.011), whereas in the postintervention survey, 76.2% and 22.7% (totally agreeing and agreeing, respectively) reported a change in their perspective and sensitivity toward the older population (*p*=0.015). Furthermore, 79.3% of the participants (*p*=0.029) reported a positive impact on their education and 14.5% (*p*=0.037) reconsidered pursuing a specialized degree associated with the care of older individuals after undergoing the intervention. The consequence of reconsidering pursuing a specialized or graduate degree associated with the care of the older population was more evident among the participants with earlier knowledge (aged 18–20 years) regarding senescence and the professional care of older people as opposed to the other age groups (older than 20 years; *p*=0.01), which was a significant finding in this study.

Conversely, we determined that nutrition and psychology students profile were more aware of the fall risk in the older population than medical and nursing students (34.8% and 32.8%, respectively, *p*=0.001) in the analysis by the professional area group. Similarly, nutrition, psychology, and nursing students stated that the health system is not adequately efficient in meeting the needs of the older population as opposed to the medical, radiology, and physical education students (*p*=0.008).

## 4. Discussion

Designing a simulator to create an experiential educational strategy to increase the knowledge and self-perception related to the elderly has been the most relevant challenge in educating and raising sensitivity regarding the care of older population.

The current study comprised several stages, one of the most important being educational interventions by way of informative sessions in health sciences for the elderly. At this stage, the complementary application of this strategy in real time through an experiential essay contributes to sensorially feel the changes present in the evolution of senescence, representing a transcendent educational opportunity for the development of empathy as a central axis of health care. Audiovisual and digital technologies had to be developed during the pandemic stage to conduct this strategy virtually as well.

By designing the abovementioned strategy and applying it to students from different areas associated with the field of health sciences in a random fashion, we could monitor the project and assess the impact of this educational intervention using semistructured preintervention and postintervention surveys, the responses of which were statistically analyzed, according to other authors [27, 28].

Some of the most relevant factors that were assessed included the perception of and sensitivity toward the older population, the impact of the intervention on the participants, future professional vision, the knowledge, attitude, and the possibility of the participants pursuing graduate degrees in fields associated with the study, assistance, and rehabilitation of older adults [29–34].

When analyzing the health context perception and services provided to the older population, most participants described the health system as deficient and required further improvement to enhance its perspective of and efficiency toward caring for the older population who are considered vulnerable. This applies to the quality of health sciences education in this field, which was described as adequate by 59% of the participants.

In the comparative analysis, increased awareness regarding the physiological limitations of the older population and an increased perception of sensitivity toward them (98.9%) was observed. Similarly, the participants considered that the experience of the intervention positively affected their perception regarding professionalism in the care of the older population.

These findings encourage changes in behavior of students, which are reflected by the fact that 14.5% of the participants stated they would reconsider pursuing a degree associated with the care of the older population. This proportion is higher in the younger participants, i.e., in the 18–20 years age group, as opposed to the group of students over the age of 20 years (*p*=0.01). Finally, 90.2% of the participants described the intervention as beneficial and relevant to the curricular models.

Assessing the attitude and behavior changes through new methodologies highlights the idea of developing models with a deeper effect on curricular and professional education for the management of the older population [32–41].

In educational aspects, this strategy generates knowledge related to senescence, demonstrates the level of perception of the needs of patients with functional limitations, and contributes to promote more empathetic behaviors in the management of these cases.

### 4.1. Study Limitations

All the participants could not physically wear the simulator due to logistic and time-related reasons. Despite sharing the same study objectives and variables, the preintervention and postintervention survey questions did not have the same formulation in the preevaluation and postevaluation, thereby limiting the possibility of conducting wider comparative statistical analyses between the groups. Indeed, an observational/simulation-based approach study would be more appropriate, but the lack of simulator equipment to dress each and every participant limited this possibility. The qualitative variables could be better evaluated through a different, more specific methodology to capture the certainty of self-perception.

## 5. Conclusions

The findings of this study confirm the importance of considering other alternatives within the health sciences education field and their effect on the proactive processes and behavior changes, knowledge, and attitudes of the individuals practicing in this domain. Educational strategies, such as the senescence simulator, offer an experiential intervention that strengthens the knowledge and attitudes toward older individuals. During the pandemic emergency, it proved to be a useful educational strategy in consolidating caring behavior as a hybrid educational tactic. The senescence simulation enabled the participants to widen their educational and professional schemes to encompass the care of the older population.

## Figures and Tables

**Figure 1:** Design, components, and functionality of the senescence simulator.

**Table 1:** Results of the preintervention survey.

Survey elements	Results (*n* = 256)
Demographic data	
Sex	
Women	178 (69.5%)
Men	78 (30.5%)
Age (mean (SD))	21.2 (3.1)
Degree	
Physical education and sports	13 (5.1%)
Nursing	65 (25.4%)
Medicine	82 (32%)
Nutrition	23 (9%)
Psychology	61 (23.8%)
Radiology	12 (4.7%)
The participant has considered pursuing a specialized or graduate degree	
Yes	216 (84.4%)
No	2 (0.8%)
Maybe	38 (14.8%)
Study area that the participant would likely choose for the specialized or graduate degree	
Pediatric care	77 (30.1%)
Adolescence care	31 (12.1%)
Adult care	121 (47.3%)
Older population care	27 (10.5%)
Prior experience in the care of an older adult	
Yes	141 (55.1%)
No	115 (44.9%)
Knowledge regarding the approximate annual fall rate among the older population	
Correct answer^a^	70 (27.3%)
Incorrect answer	107 (41.8%)
Does not know	79 (30.9%)
Knowledge regarding the main disabilities among the older population^b^	
Cognitive deterioration	240 (93.8%)
Osteoporosis	223 (87.1%)
Kyphosis	123 (48%)
Peripheral neuropathy	180 (70.3%)
Neurogenic claudication	82 (32%)
Cataracts	216 (84.4%)
Urinary incontinence	210 (82%)
Presbycusis	196 (76.6%)
Cervical spondylosis	126 (49.2%)
Decreased motor skills	214 (83.6%)
Balance alterations	192 (75%)
The participant considers that the current health system satisfactorily meets the needs of the older population	
Totally agrees	2 (0.8%)
Agrees	12 (4.7%)
Neutral response	67 (26.2%)
Disagrees	136 (53.1%)
Totally disagrees	39 (15.2%)
The participant considers that caregivers are adequately trained to care for the older population and meet their needs	
Totally agrees	84 (32.8%)
Agrees	46 (18%)
Neutral response	87 (34%)
Disagrees	34 (13.3%)
Totally disagrees	5 (2%)
According to the participant, the biggest problem that the older population faces is …	
Discrimination	12 (4.7%)
Intolerance	92 (35.9%)
Violence	10 (3.9%)
Abandonment	142 (55.5%)

^a^Correct answer: 1 out of every 4 older adults [9]. ^b^The terms used in the survey have been adapted for the general public to ensure a better understanding.

**Table 2:** Results of the postintervention survey.

Survey elements	Answers (*n* = 256)					
The participant is aware regarding the limitations faced by the older population that were mentioned in the educational session						
Yes	32 (12.5%)					
No	22 (8.6%)					
Only some	202 (78.9%)					

	Totally agrees	Agrees	Neutral response	Disagrees	Totally disagrees	Not applicable
The participant's perception changed; empathy and understanding toward the physical and cognitive limitations of the older population increased	195 (76.2%)	58 (22.7%)	3 (1.2%)	0 (0%)	0 (0%)	
The intervention positively affected the participant's professionalism in providing better care for the older population	203 (79.3%)	52 (20.3%)	1 (0.4%)	0 (0%)	0 (0%)	
The participant's manner of care and management for the older population will change (only for the participants with prior experience in older population care)	142 (55.5%)	42 (16.4%)	2 (0.8%)	1 (0.4%)	0 (0%)	69 (27%)
The participant has reconsidered pursuing a specialized or graduate degree associated with the care of the older population	37 (14.5%)	87 (34%)	92 (35.9%)	32 (12.5%)	8 (3.1%)	
The participant considers that the education provided in his/her educational institution regarding the care of the older population is adequate	89 (34.8%)	64 (25%)	59 (23%)	40 (15.6%)	4 (1.6%)	
The participant considers that the use of a simulation-based exoskeleton is relevant for his/her education	137 (53.5%)	94 (36.7%)	23 (9%)	2 (0.8%)	0 (0%)	

**Table 3:** Results of the main variables assessing the effect of the educational intervention in students in terms of their degree.

Survey element	Degree	Totally agrees	Agrees	Neutral response	Disagrees	Totally disagrees
The participant's perception changed; empathy and understanding toward the physical and cognitive limitations of the older population increased	Psychology	70.5	27.9	1.6	0	0
	Medicine	80.5	18.3	1.2	0	0
	Nursing	78.5	20	1.5	0	0
	Nutrition	78.3	21.7	0	0	0
	Physical culture and sports	61.5	38.5	0	0	0
	Radiology	75	25	0	0	0

The intervention positively affected the participant's professionalism in providing better care for the older population	Psychology	67.2	32.8	0	0	0
	Medicine	85.4	13.4	1.2	0	0
	Nursing	84.6	15.4	0	0	0
	Nutrition	82.6	17.4	0	0	0
	Physical culture and sports	61.5	38.5	0	0	0
	Radiology	83.3	16.7	0	0	0

The participant has reconsidered pursuing a specialized or graduate degree associated with the care of the older population	Psychology	8.2	34.4	39.3	18	0
	Medicine	6.1	35.4	41.5	13.4	3.6
	Nursing	23.1	29.2	33.8	12.3	1.5
	Nutrition	21.7	43.5	21.7	4.3	8.7
	Physical culture and sports	30.8	23.1	38.5	7.7	0
	Radiology	25	41.7	16.7	0	16.7

Values are presented as percentages.

## Data Availability

The experimental data and results supporting the conclusions of this study are publicly available in the Figshare repository with the identifier: https://doi.org/10.6084/m9.figshare.22597249.
